RETRACTED

# U-Net-Based Medical Image Segmentation

**DOI:** 10.1155/2022/4189781

**Published:** 2022-04-15

**Authors:** Xiao-Xia Yin, Le Sun, Yuhan Fu, Ruiliang Lu, Yanchun Zhang

**Affiliations:** ^1^Cyberspace Institute of Advanced Technology, Guangzhou University, Guangzhou 510006, China; ^2^College of Engineering and Science, Victoria University, Melbourne, VIC 8001, Australia; ^3^Engineering Research Center of Digital Forensics, Ministry of Education, Nanjing University of Information Science and Technology, Nanjing, China; ^4^Department of Radiology, The First People's Hospital of Foshan, Foshan 528000, China

## Abstract

Deep learning has been extensively applied to segmentation in medical imaging. U-Net proposed in 2015 shows the advantages of accurate segmentation of small targets and its scalable network architecture. With the increasing requirements for the performance of segmentation in medical imaging in recent years, U-Net has been cited academically more than 2500 times. Many scholars have been constantly developing the U-Net architecture. This paper summarizes the medical image segmentation technologies based on the U-Net structure variants concerning their structure, innovation, efficiency, etc.; reviews and categorizes the related methodology; and introduces the loss functions, evaluation parameters, and modules commonly applied to segmentation in medical imaging, which will provide a good reference for the future research.

## 1. Introduction

Interpretation of medical images such as CT and MRI requires extensive training and skills because the segmentation of organs and lesions needs to be performed layer by layer. Manual segmentation means a heavy workload to the doctors, which can introduce bias if it involves the subjective opinions of doctors. To analyze complicated images, it usually requires doctors to make a joint diagnosis, which is time consuming. Furthermore, automatic segmentation is a challenging task, and it is still an unsolved problem for most medical applications due to the wide variety connected with image modalities, encoding parameters, and organic variability.

According to [1], medical imaging increased rapidly from 2000 to 2016. As illustrated in Figure 1(a), retrospective cohort study of patterns of medical imaging between 2000 and 2016 was conducted among 16 million to 21 million patients. These patients were enrolled annually in 7 US integrated and mixed-model insurance health care systems and for individuals receiving care in Ontario, Canada. Relative imaging rates by different imaging modality, such as computed tomography (CT), magnetic resonance imaging (MRI), and ultrasound that are used by adults [18–64 years] annually in US and Ontario are also illustrated in Figures 1(b)–1(d), respectively. The imaging rates (per 1000 people) of CT, MRI, and ultrasound use continued to increase among adults, but at lower pace in more recent years. Whether the observed imaging utilization was appropriate or was associated with improved patient outcomes is unknown.

RETRACTED

Nowadays, the application of deep learning technology in medical imaging has attracted extensive attention. How to automatically recognize and segment the lesions in medical images has become one of the issues that concern lots of researchers. Ronneberger et al. [2] proposed U-Net at the MICCAI conference in 2015 to tackle this problem, which was a breakthrough of deep learning in segmentation of medical imaging. U-Net is a Fully Convolutional Network (FCN) applied to biomedical image segmentation, which is composed of the encoder, the bottleneck module, and the decoder. The widely used U-Net meets the requirements of medical image segmentation for its U-shaped structure combined with context information, fast training speed, and a small amount of data used. The structure of U-Net is shown in Figure 2.

Containing many slices, biomedical images are often blocky in a volume space. An image processing algorithm of 2D is often used to analyze a 3D image [3–7]. But when the information is sorted and trained one by one, it would result in increased computational expenses and low efficiency. Therefore, it is difficult to deal with volume images in many cases. A 3D U-Net model derived from the 2D U-Net is designed to address these problems. To further target on architectures of different forms and dimensions, Oktay et al. [8] proposed a new attention gate (AG) model for medical imaging analysis. The model trained with AG indirectly learns to restrain irrelevant regions in an input image and highlight striking features suitable for specific tasks. This is conducive to eradicating the inevitability of applying overt exterior tissue/organ localization units of cascading convolutional neural networks (CNNs) [8, 11]. AG could be combined with standard CNN structure like U-Net, which increases the sensitivity and the precision of the model. To get more advanced data and retain spatial data aimed at 2D segmentation, Gu et al. in 2019 [12] proposed the context encoder network (CE-Net), using pretrained Res-Net blocks as fixed feature extractors. It is mainly composed of three parts—feature encoder, context extractor, and feature decoder. The context extractor is composed of a newly introduced dense atrous convolution (DAC) block and a residual multikernel pooling block (RMP). The introduced CE-Net is widely applied to segmentation in 2D medical imaging [11] and outperforms the original U-Net method.

RETRACTED

To further advance the segmentation, UNet++, a novel and greater neural network structure for image segmentation was proposed by Zhou et al. [13]. Moreover, it is a deeply supervised encoder-decoder network connected by a series of nested and dense hopping paths to narrow the semantic gap between the encoding and decoding subnetwork feature maps. Later, to improve more accuracy, especially for organs of different sizes, a new version UNET 3+ was designed by Huang et al. [14]. It utilizes full-scale skip links and deep supervisions, which combines low-level details and high-level semantics mapped at different scales of features and learns hierarchical representation from full-scale aggregated feature maps. The suggested UNet 3+ could increase computational productivity by decreasing network parameters.

Framework regarding nnU-Net (“no-new-Net”) is developed by Isensee et al. [15] as a robust self-adaptive framework from U-Net. It was designed by making slight alterations to the 2D and 3D U-Net, where 2D, 3D, 2D, and 3D links were proposed to work together and form a network pool. The nnU-Net could not only automatically adapt its architecture to the given image geometry, but thoroughly define all the other steps including image preprocessing, data training, testing, and potential postprocessing.

U2-Net as a simple and powerful deep network architecture developed by Qin et al. [16] consists of a two-level nested U-shaped structure applied to salient target detection (SOD). It has the following advantages: (1) due to the mixed receptive fields of various sizes in the proposed residual U-shaped block (RSU), it could capture a larger amount of contextual data at various scales. (2) The pooling operation used in the RSU block increases the depth of the entire structure without substantially pushing up the computational cost.

TransUNet designed by Chen et al. [17] encodes tokenized image patches and extracts global contexts from the input sequence of CNN feature map; the decoder upsamples the encoded features and combines with the high-resolution CNN feature maps for precise localization. It uses transformers as a powerful encoding structure for segmentation. Due to the inherent locality of convolution operations, U-Net usually shows limitations in clearly modeling dependencies. The transformer designed for sequence-to-sequence prediction has become an alternative architecture with an innate global self-attention mechanism while localization capabilities of the transformer frame may be limited due to insufficient low-level details.

Since U-Net was proposed, its encoder-decoder-hop network structure has inspired a large amount of segmentation means in medical imaging. Such deeplearning technologies as attention mechanism, dense module, feature enhancement, evaluation function improvement, and other basic U-Net structures have been introduced into medical image segmentation and become widely adopted. These variations of U-Net-related deep learning networks are designed to optimize results by improving the accuracy and computing efficiency of medical image segmentation through changing network structures, adding new modules, etc. However, most of the existing literature related to U-Net focused on introducing isolated new ideas and rarely gave a comprehensive review that summarizes the variations of the U-Net structure for deep learning of segmentation in medical imaging. This paper discussed some of these ideas in more depth.

RETRACTED

To sum up, the basic motivation behind this work is not to elaborate into new ideas in U-Net-related deep learning networks but to use effectively U-Net-related deep learning networks techniques into the segmentation of multidimensional data for biomedical applications. The presented method can be generalized to any dimension and can be used effectively to other types of multidimensional data as well.

This paper is organized as follows.  Section 2 addresses the current challenges faced by medical image segmentation.  Section 3 reviews these variations of U-Net-related deep learning networks.  Section 4 collects various experiment results in literature in relation to different U-Net networks, along with the validation parameters for optimized network structure through the associated deep learning models. The future development in the U-Net-based variant networks is analyzed and discussed. Finally, Section 5 concludes this paper.

## 2. Existing Challenges

This section presents the current challenges faced by medical image segmentation which make it inevitable to improve and innovate U-Net-based deep learning approaches.

First, medical image processing requires extremely high accuracy for disease diagnosis [18–23]. Segmentation in medical imaging refers to pixel-level or voxel-level segmentation. Generally, the boundary between multiple cells and organs is difficult to be distinguished on the image [3]. Moreover, the data obtained from the image are usually preprocessed, the relevant network is built, which continues to be run by adjusting the parameters even though a certain level of accuracy is reached by using the relevant deep learning model [24].

Second, medical images are acquired from various medical equipment and the standards for them and annotations or performance of CT/MRI machines are not uniform. Hence deep-learning-related trained models are only suitable for specific scenarios. Meanwhile, the deep network with weak generalization may easily capture wrong features from the analyzed medical images. Furthermore, significant inequality always exists between the size of negative and positive samples, which may have a greater impact on the segmentation. However, U-Net could afford an approach achieving better performance in reducing overfitting [25].

RETRACTED

Third, interpretable deep learning models applied to analyze medical images are highly required, but there is a lack of confidence in its predicted results [26, 27]. U-Net is a CNN showing poor interpretability. Segmentation in medical imaging could reflect the patient's physiological condition and accurate disease diagnosis. It is not easy for the segmentation lacking interpretability and confidence to be trusted and recognized by professional doctors for clinic application. Although disease diagnosis mainly relies on images, combined with other supplements, which has also increased the complexity. It is a challenge to realize the interpretability and confidence of medical image segmentation via perceiving and adjusting these trade-offs.

## 3. Methodology

Various medical image segmentation methods have been developed very quickly based on U-Net for performance optimization. U-Net is improved in the areas of application range, feature enhancement, training speed optimization, training accuracy, feature fusion, small sample training set, and generalization improvement. Various strategies are applied in the designing of different network structures to address different segmentation problems.

This section is focused on variations of U-Net-based networks, with the description of U-Net framework, followed by the comprehensive analysis of the U-Net variants by performing (1) intermodality and (2) intramodality categorization to establish better insights into the associated challenges and solutions. The main related work is summarized from the aspects of the improved performance indicators and the main structural characteristics.

### 3.1. Traditional U-Net

The traditional U-Net is two-dimensional network architecture whose structure is shown in Figure 2. U-Net modifies and extends the Fully Convolutional Network (FCN), making it work with very few training images and produce more accurate segmentation. The major idea is to replace the general shrinkage network with sequential layers and the pooling operation is related to downsampling operator, which is supplemented by upsampling operator. Hence the output's resolution is raised by these layers. The high-resolution of the contracted path is combined with the upsampled output for localization. Hence sequential convolutional layers could study fine features and result in a more accurate segmentation.

RETRACTED

An important modification in the U-Net architecture lies in the upsampling section, where there are huge amounts of feature channels allowing the network to spread contextual data to higher-resolution layers. Therefore, the expansion path is roughly symmetrical to the contraction path, forming a U-shaped structure. The network applies the effective part of every convolution—the map of segmentation contains mere pixels, and the complete context of the pixels could be obtained in the input image. This method allows seamless segmentation in arbitrarily large imaging using crucial overlapping tiling strategies, without which the resolution will be limited by GPU memory [1].

The traditional CNN is usually connected to several fully connected layers after convolution and the feature map produced by the convolutional layer is mapped into a feature vector with a fixed length for image-level classification. An improved FCN structure, however, identifies the image at the pixel level, thereby facilitating the task of segmentation in imaging at the semantic level [28].

U-Net could be applied to the segmentation due to its large measurement size of medical images. It is impossible to input the large medical images into the network when they are segmented and required to be cut into small pieces. Overlapping-tilling strategies are suitable for small pieces cutting using U-Net due to its network structure. Thus, it could accept images of any size as inputs [29].

### 3.2. 3D U-Net

Biomedical imaging is a set of three-dimensional images composed of slices at different locations. Biomedical image analysis involves dealing with a large amount of volume data. Annotating these data labeled by segmentation could cause difficulties because only two-dimensional slices can be displayed on computers. Therefore, low efficiency and loss of contexts are common during 3D-image processing by traditional 2D image models. To solve this, Ozgun Cicek et al. [30] put forward a 3D U-Net with a shrinking encoder part for analyzing the entire image and a continuous expansion decoder part for generating full-resolution segmentation on the basis of the previous U-Net structure. The structure of 3D U-Net is similar to 2D U-Net in many aspects, except that all operations in the 3D network are replaced with corresponding 3D convolution, 3D pooling, and 3D upsampling. Batch normalization (BN) [31] is used to prevent the network bottlenecks.

Just like the standard U-Net, there is an encoding path and a decoding path with 4 parsing steps in every layer in the encoding path. It contains two 3 × 3 × 3 convolutions followed by a corrected linear unit (ReLu) and then a 2 × 2 × 2 maximum pooling layer with 2-step size of each. Every layer in the synthesis path is composed of 2 × 2 × 2 upper convolutions with two steps in each dimension and two subsequent 3 × 3 × 3 convolutions with a ReLu active layer behind each. The skip connections from the equal-resolution feature map in the encoding path provide the necessary high-resolution features for the decoding path. In the last layer, 1 × 1 × 1 convolution decreases the quantity of output channels to that of labels standing at 3. The structure has 19069955 parameters in total.

RETRACTED

In addition to the rotation, scaling, and gray value increase, smooth dense deformation fields are applied to the data and ground truth labelers before training Therefore, random vectors are sampled from a general distribution whose standard deviation is 4 in a grid spaced 32 voxels in each direction, followed by the application of B-spline interpolation. The softmax with weighted cross-entropy loss is used to compare the network output and the ground truth label, to reduce the weight of the common background, increase the weight of internal tubules, and realize the balance effect of small blood vessels and background voxels on the loss.

This end-to-end learning strategy could use semiautomatic and completely automatic methods to segment 3D targets from sparse annotations. The structure and data enhancement of this network allow it to learn from a small number of labeled data and to obtain good generalization capabilities. Appropriate rigid transformation and minor elastic deformation applications could generate reasonable images, rationalize its preprocessing method, and enable the network structure to be extended to any size of the 3D data set.

### 3.3. Attention U-Net

Attention could be considered as a method of organizing computational resources to interpret the signal informatively. Since its introduction, the attention mechanism has become more and more popular in the deep learning industry. This paper summarizes a method in the application of the attention mechanism onto the U-Net network. Given the small lesions and large shape changes, the attention module is generally added in image segmentation before the encoder- and decoder-related features are stitched or at the bottleneck of U-Net to reduce false-positive predictions.

The Attention U-Net put forward by Oktay et al. [8] in 2018 adds an integrated attention gate (AG) before U-Net splices the corresponding features in the encoder and decoder and readjusted the output features of the encoder. This module facilitates generation of gating signal to eliminate the response of irrelevant and noisy ambiguity in the skip connection, emphasizing the salient features transmitted via the skip connection. Figure 2 displays the inside structure of the attention module.

RETRACTED

The salient features useful for specific tasks are stressed in the model trained by AG, which indirectly learns and suppresses unconcerned areas of the input image. Thus, obvious exterior tissue/organ positioning modules are not necessarily used in the Cascaded CNN. Without extra computational cost, the forecast precision and sensitivity of the model could be improved by AG due to its compatibility in standard CNN architectures like U-Net. To estimate the attention U-Net structure, two big CT abdominal data sets were used for multiclass segmentation in imaging. The results show a significant enhancement of U-Net's prediction performance by AG under different data sets and training scales, and the computational efficiency is maintained as well.

The structure of attention U-Net, as shown in Figure 3, is a U-Net-based structure with two stages: encoding and decoding. The coarse-grained map of the left structure captures information in the context and highlights the type and position of foreground objects. Subsequently, feature maps extracted from numerous scales are fused via jump links to merge coarse-grained and fine-grained dense predictions. As for the method put forward in the paper, the attention gate mechanism is to add an AG to each skip connection layer to spread the attention coefficient. AG has two inputs, *x* from the feature map of the shallow network on the left and *g* from that of the lower network, which will be output from AG. Then the feature fusion is performed on the feature map after sampling on the right.

This method makes it unnecessary to utilize external object positioning models. It is a convenient tool not only used in natural image analysis and machine translation but also in image classification and regression. Studies showed that the algorithm is very useful for the identification and positioning of tissues/organs, and a certain degree of accuracy could be achieved in the use of smaller computing resources, especially for small-sized organs such as the pancreas [32].

### 3.4. CE-Net

A fusion of features with different scales serves as a crucial approach to optimizing segmentation performance. Due to fewer convolutions, the low-level features experience lower semantics and more noise despite of their higher resolution and more position. In addition, the resolution is considerably low and the detail perception is poor despite that high-level features contain more intensive semantic information. It is of huge significance to efficiently combine the advantages of these two to improve the segmentation model. Feature fusion includes the contextual features' fusion of the network and the fusion of different modal features in a larger sense. Gu et al. [10] designed a new network called CE-Net, which adopts new modules of dense atrous convolution block (DAC) and residual multikernel pooling block (RMP) to offer fused information like the fusion of contextual features from the encoder, to get higher-level information with a decrease in the feature loss [33], for example, to retain spatial information for 2D segmentation in medical imaging and classification [34].

RETRACTED

The overall framework of CE-Net is shown in Figure 4. The DAC block could identify broader and more in-depth semantic features via injecting four cascaded branches with multiscale dense hole convolution. The remaining connections are used to prevent the gradient from disappearing. In addition, the RMP block is a residual multicore pool based on the spatial pyramid pool, which encodes the multiscale context features of the object extracted from the DAC module without extra learning weights using various size pool operations. In summary, the DAC block extracts rich feature representations through multiscale dense hole convolution and then uses the RMP block to extract more context information through multiscale pooling operations. The joint use of newly proposed DAC block and RMP block with the backbone codec structure is unprecedented in CE-Net's context encoder network. This allows the enhancement of the segmentation by further collecting abstract features and maintaining more spatial information.

#### 3.4.1. Feature Encoder Module

In the U-Net structure, each encoder block includes two convolutional layers and a maximum pooling layer. As for the CE-Net network structure, a pretrained ResNet-34 is used in the feature encoding module and the first four feature extraction blocks are retained without mean pooling and full connection. Res-Net adds a shortcut mechanism to avoid gradient disappearance and improve the network convergence efficiency, as shown in Figure 4(b). It is a basic method to improve U-Net segmentation performance using pretrained Res-Net.

#### 3.4.2. Context Extraction Module

The context extraction module, composed of DAC and RMP, extracts contextual semantic information and produces more advanced feature maps.

*(1) Hollow Convolution*. As for semantic segmentation and object detection, deep convolutional layers have displayed superiority in image feature representation extraction. But the pooling layer might cause loss of image semantic information, which is solved by applying dense hole convolution [35] to dense image segmentation. The hole convolution has an expansion rate parameter which implies that the size of the expansion and the convolution kernel is the same with the ordinary convolution. It means parameters remain unchanged in the neural network, but the hole convolution has a larger receptive field, which refers to the size involved by the convolution kernel on the image. The size of the receptive field is related to stride, the number of convolutional layers, and padding parameters.

*(2) DAC*. Inspired by Inception [36, 37], Res-Net [38], and hole convolution, dense hole convolution blocks (DAC) [11] are used for encoding high-level semantic feature maps. The DAC has four branches cascading down, with the acceptance field of each branch being 3, 7, 9, and 19, respectively and a gradual increase in the number of atrous convolutions. DAC uses different receptive fields like the inception structure. In each hole convolution branch, a 1 × 1 convolution is applied to ReLu. The shortcut links in Res-Net are used directly to add the original features. Generally, the convolution of the large receptive field could extract and produce a larger number of abstract features for the large target and vice versa. The DAC block can extract features from the targets of various sizes through the combination of hole convolutions and different expansion rates.

*(3) RMP*. One of the challenges in medical image segmentation lies in the significant change in target size [39, 40]. For instance, an advanced tumor is usually much bigger than the early one [41]. An RMP [11] is proposed to solve this problem, by which targets with various sizes could be detected by applying numerous effective fields of view. The proposed RMP utilizes four receptive fields with different size to encode global context information. To reduce the dimensionality of the weights and the computational cost, a 1 × 1 convolution is used after each pooling branch. Afterwards, the upsampling of the low-dimensional feature map is performed to obtain the same size of features as an original feature map through bilinear interpolation, allowing extraction of features of various scales.

RETRACTED

#### 3.4.3. Feature Decoder Module

The feature decoder module allows the recovery of the high-level semantic features extracted from the context extractor module and the feature encoder module. Continuous pooling and convolution operations often lead to the loss of information, which, however, can be remedied by conducting a quick connection from the encoder to the decoder. In U-shaped networks, the two basic operations of decoder are simple upsampling and deconvolution. The image can be enlarged by conducting upsampling through linear interpolation. Deconvolution (also known as transposed convolution) uses convolution to expand the image. Adaptive mapping is used in transposed convolution to recover more comprehensive information. Therefore, transposed convolution is implemented to achieve a higher resolution in the decoder. Based on the shortcut connection and the decoder block, the feature decoder module produces a mask of the same size as the original input.

Unlike U-Net, CE-Net applies a pretrained Res-Net block in the feature encoder. The integration of DAC module, RMP module and Res-Net into the U-Net architecture allows it to retain more spatial information. It was suggested that this approach could optimize segmentation in medical imaging for various tasks of optic disc segmentation [42], retinal blood vessel detection [11], lung segmentation [11], cell contour segmentation [35], and retinal OCT layer segmentation [43]. This approach could be extensively utilized in other 2D medical image segmentation tasks.

### 3.5. UNET++

Variants of encoder and decoder architectures such as U-Net and FCN are found to be the most advanced image segmentation models [44]. These segmentation networks share a common feature—skip connections that link the depth, semantics, and coarse-grained feature maps from the decoder subnetwork together with the shallow, low-level, and fine-grained feature mapping from the encoder subnetwork. More pinpoint precision is needed in segmentation of lesions or abnormalities in medical images needs than regular images. Edge segmentation faults in medical imaging may cause some serious consequences in clinic. Therefore, a variety of methods to improve feature fusion have been proposed to address that. In addition, Zhou et al. [13, 45] improved the skip connection and proposed UNet++ with deep monitoring nested dense jump connection path.

As for U-Net, the feature map of the encoder is received by the decoder. But UNet++ uses a dense convolutional block and the quantity of convolutional layers relies on that of the U-shaped structure. In essence, the dense convolution block connects the semantic gap between the encoder and decoder feature maps. It is assumed that when the received encoder feature map and the related decoder feature map are similar at the semantic level, the optimizer can easily tackle the problems it encounters. The effective integration of U-Nets of different depths is used to alleviate unknown network depths. These U-Nets could share an encoder in part and simultaneously learn together through deep supervision, which will allow the model to be pruned and improved. This redesigned skip connection could aggregate semantic features of different scales on the decoder subnet, thereby automatically generating a highly flexible feature fusion scheme.

RETRACTED

### 3.6. UNET 3+

UNet++, an improvement based on U-Net, was designed by developing a structure with nested and dense skip connections. But it does not express enough information from multiple scales and the network parameters are numerous and complex. UNet 3+ (UNet+++) is an innovative network structure proposed by Huang et al. [46], which uses full-scale skip connections and deep supervisions. Full-scale jump connection combines high-level semantics with low-level semantics from feature maps of various scales. Deep supervision learns hierarchical representations from feature maps aggregated at multiple scales. This method uses the newly proposed hybrid loss function to refine the results, particularly suitable for resolving organs of different sizes. It not only improves accuracy and computational efficiency, but also reduces network parameters after fewer channels compared to U-Net and UNet++. The network structure of UNet 3+ is shown in Figure 5.

To learn hierarchical representation from full-scale aggregated feature maps, UNet 3+ further adopts full-scale deep supervision. Different from UNet++, each decoder stage in UNet 3+ has a side output, which uses standard ground truth for supervision. To achieve in-depth supervision, the last layer at each decoder stage is sent to an ordinary 3 × 3 convolutional layer, followed by a bilinear upsampling and a sigmoid function to enlarge it to full resolution.

To further strengthen the organ's boundary, a multiscale structural similarity index loss function is proposed to give more weight to the fuzzy boundary. Facilitated by this, UNet 3+ will focus on fuzzy boundaries. The more significant the difference in regional distribution is, the greater the MS-SSIM value becomes [47].

In segmentation of most nonorgan images, false positives are inevitable. The background noise information most likely stays at a shallower level, causing oversegmentation. UNet3++ solves this problem by adding classification-guidance module (CGM) designed to foresee whether the input image has organs to realize more accurate segmentation. With the largest number of semantic information, the classification results could further direct each segmentation side to be output in two steps. With the help of the argmax function, the two-dimensional tensor is converted into a single output of {0, 1}, which represents the presence/absence of organs. Subsequently, the single classification output is multiplied with the side segmentation output. Given the simplicity of the binary classification task, this module could easily obtain accurate classification by optimizing the binary cross-entropy loss function [48] and realize the direction of oversegmentation of nonorgan images.

RETRACTED

In summary, UNet 3+ maximizes the application of full-scale feature maps and achieves precise segmentation and efficient network structure with fewer parameters and deep supervision. It has been extensively validated, for example, on representative but demanding volumetric segmentation in medical imaging: (i) liver segmentation from 3D CT scans and (ii) whole heart and big vessels segmentation from 3D MR images [49]. The CGM and the hybrid loss function are further applied to obtain a higher level of accuracy in location-aware and boundary-aware segmented images.

### 3.7. nnU-Net

It has been designed for different tasks since U-Net was first proposed, with its different network structure, preprocessing, training, and inference. These options are dependent on each other and significant to the final result. Fabian et al. [15, 50] proposed nnU-Net, namely no new-Net. The network is based on 2D and 3D U-Net with a robust self-adaptive framework. It involves a set of three relatively simple U-Net models. Only slight modifications are made to the original U-Net, and no various extension plug-ins were used, including residual connection, dense connection, and various attention mechanisms. The nnU-Net gives unexpectedly accurate results in applications like accurate brain tumor segmentation [51]. Since medical images are often three-dimensional, the design of nnU-Net considers a basic U-Net architecture pool composed of 2D U-Net, 3D U-Net, and U-Net cascade. 2D and 3D U-Net could generate full-resolution results. The first stage of the cascaded network produces a low-resolution result and the second stage optimizes it.

Now that 3D U-Net is widely used, why is 2D still useful? This is because the author proves that when the data are anisotropic, the traditional 3D segmentation method becomes very poor in resolution. The 3D network takes up a lot of GPU memory. Then you could use smaller image slices for training, but for images of larger organs such as livers, this block-based method will hinder training. This is caused by the limited size of the receptive field; the network structure cannot collect enough contextual information to identify the target objects. A cascade model is used here to overcome the shortcomings of 3D U-Net on data sets with large image size. First, the first-level 3D U-Net is trained on the downsampled image and afterward the result is upsampled to the original voxel interval arrangement. The upsampling result is sent to the second-level 3D U-Net as an additional input channel (one-hot encoding) and the image block-based strategy is used for training on the full-resolution image.

RETRACTED

The structure of U-Net has negated most of the new network structures in recent years. It is believed that the network structure has been advanced. The more complex the network, the greater the risk of overfitting. More attention should be paid to other factors such as preprocessing, training, reasoning strategies, and postprocessing.

### 3.8. U2-Net

Salient object detection (SOD) [52] was designed to segment the most visually attractive objects in the image. It is extensively applied to eye-tracking data [53], image segmentation, and other fields. The recent years have seen a progress in deep CNN especially the emergence of FCN in image segmentation, which substantially enhances the performance of salient target detection. Most SOD network designs share a common pattern, which is to focus on the application of deep features extracted from the present backbone networks, e.g., AlexNet [54, 55], VGG [56], Res-Net [57], ResNeXt [39, 58], and DenseNet [59]. But these backbone networks were proposed for image classification, which extract features that represent semantics instead of local details and global contrast information that are crucial for saliency detection. They must pretrain on the data-inefficient ImageNet data, especially when the target data follows a different distribution from ImageNet.

U2-Net [16, 60] is an uncomplicated and powerful deep network used for salient target detection. It does not use a pretrained backbone model for image classification and could receive training from scratch. It could capture more contextual information because it uses the RSU (ReSidual U-blocks) structure [60, 61], which combines the characteristics of different scales of receptive fields. Meanwhile, it enhances the depth with entire architecture but without significantly increasing computational cost when the pooling operations are applied to these RSU blocks.

*RSU structure*: as to SOD and other segmentation tasks, both local and global context information is of great significance. As to modern CNN designs, VGG, Res-Net, DenseNet, 1 × 1 or 3 × 3 small convolution filters are the most commonly used feature extraction components. Despite its high computational efficiency and small storage size, its filter experience is too small to capture global information; hence, the shallow output feature map only contains local features. To obtain more global information on the shallow high-resolution topographic map [62, 63], the most direct method is to expand the receiving field.

The existing convolutional block with the smallest receptive field fails to obtain global information, and the output feature map at the bottom layer only contains local features. To obtain richer global information on high-resolution shallow feature maps, the receptive field must be expanded. There are attempts to expand the receptive field by using hole convolution to extract local and nonlocal features. However, performing multiple extended convolutions on the input feature map of the original resolution (especially in the initial stage) requires a large amount of computing and memory resources. Inspired by U-Net, a new RSU is proposed to obtain multiscale features within the stage. RSU is mainly composed of three parts as follows.

1. Input convolutional layer: convert the input feature map x(*H* × *W* × *C*_in_) into an intermediate image *F*_1_(*x*) with the number of *C*_out_ channels to extract local features.
2. Use the intermediate feature map *F*_1_(*x*) as input and learn to extract and encode multiscale context information *U*(*F*_1_(*x*)). U refers to U-Net. The greater the *L*, the deeper the RSU and the more pooling operations, the bigger the receptive field and the more local and global features.
3. Through the summation of *F*_1_(*x*), local features and multiscale features are merged.

RETRACTED

Hence the residual U-block RSU about how to stack and connect these structures is proposed. It results in a completely different method from previous cascade stacking: Un-Net. The exponential notation here means a nested U-shaped structure rather than a cascaded stack. In theory, the index *n* could be adjusted to any positive integer to realize a single-layer or multilayer nested U-shaped structure. However, to be applied to practical applications. *n* is set to 2 to form the two-leveled U2-Net. The top layer of it is a large U-shaped structure including 11 stages with each filled with a well-configured RSU. Therefore, the nested U structure could extract the multiscale features in each stage and the multilevel features in the aggregation stage with higher efficiency. Unlike those SOD models which are built on present backbones, U2-Net is constructed on the proposed RSU block that allows training from scratch and different model sizes to be configured according to the constraints of the target environment.

### 3.9. TransUNet

Due to the inherent locality of convolution operations, U-Net is usually limited in explicitly modeling remote dependencies. Recently, the transformer designed for sequence-to-sequence prediction has emerged as an alternative architecture with a global self-attention mechanism. However, its positioning capabilities are limited by its insufficient underlying details. TransUNet with the advantages of transformer [64] and U-Net was proposed by Chen et al. [17] as a powerful alternative to medical image segmentation. This is because the transformer treats the input as a one-dimensional sequence and only focuses on modeling the global context of all stages, which results in low-resolution features and a lack of detailed positioning information. Direct upsampling to full resolution cannot effectively recover this information, which results in rough segmentation results. In addition, the U-Net architecture provides a way to achieve precise positioning by extracting low-level features and linking them to high-resolution CNN feature maps, which could adequately complement for fine spatial details. An overview of the framework is shown in Figure 6.

RETRACTED

The transformer could be used as a powerful encoder for medical image segmentation and combined with U-Net to enhance finer details and restore local spatial information. TransUNet has achieved excellent performance in multiorgan segmentation and heart segmentation. In the design of TransUNet, the issue is how to encode the feature representation directly from the decomposed image patch using the transformer.

In order to complete the purpose of segmentation, that is, to classify the image at the pixel level, the most direct method is to upsample the encoded feature map to predict the full resolution of the dense output. To restore the spatial order, the size of the coding function should first reshape the size of the image from *HW*/*P*^2^ to *H*/*P* × *W*/*P*. The next step is to use 1 × 1 convolution to decrease the channel size of the reshaped feature to the number of classes. Afterward, directly upsampling the feature map to full resolution *H* × *W* is performed to predict the final segmentation result.

In summary, TransUNet mixes CNN and transformer as an encoder and allows the use of medium and high-resolution CNN feature maps in the decoding path, hence more context information can be involved. TransUNet not only uses image features as a sequence to encode strong global context but also makes good use of low-level CNN features through a U-shaped hybrid frame design.

## 4. Overview of Validation Methods of Resultant Experiments

### 4.1. Evaluation Parameters

The several U-Net-based extended structure networks introduced above possess different improved structures and characteristics, and their effects in real-world applications vary. Therefore, this paper summarized the corresponding advantages of each by comparing the parameters. The segmentation evaluation parameters play a crucial part in the evaluation of image segmentation performance. This section mainly lists several commonly used evaluation parameters in image segmentation neural networks and illustrates the characteristics of each network in various experiments.

RETRACTED

True positive (TP), true negative (TN), false positive (FP), and false negative (FN) are mainly used to count two types of classification problems. There is no doubt that multiple categories could also be counted separately. The samples are divided into positive and negative samples.

### 4.2. Performance Comparison

The related methods proposed in this paper use almost different data sets including retinal blood vessels, liver, kidney, gastric cancer, and cell sections. The data sets used by various methods are not the same; hence, it is difficult to compare different methods horizontally. This paper listed the data sets to provide an index of data set names. The performance comparison is listed in Table 1.

### 4.3. Future Development

Medical image segmentation is a popular and developing research field. As an implementation standard of medical segmentation, the U-Net network structure has been in use and improved for many years. Although the work and improvements of U-Net in recent years have begun to solve the challenges presented in Section 2, there are still some unsolved problems. In this part, some promising research discussing those problems will be outlined (accuracy issues, interpretability, and network training issues) and other challenges that may still exist will be introduced.

#### 4.3.1. Higher Generalization Ability

The model is not only required to have a good fit (training error) to the training data set but also to have a good fit (generalization ability) to the unknown data set (prediction set). As for tasks like medical image segmentation, small sample data are usually more prone to overfitting or underfitting. Therefore, the frequently used methods such as early stopping, regularization, feedback, input fuzzification, and dropout have improved the generalization problem of neural networks to varying degrees. But in general, the essence of the neural network is instance learning and the network has the cognition of most instances through limited samples. However, recently it has been suggested to seek innovation and abandon the long-used input vector fuzzification processing method.

#### 4.3.2. Improved Interpretability

As for Interpretability or Explainable Artificial Intelligence (XAI), what always concerns researchers engaged in machine learning is that many current deep neural networks cannot fully understand the decision-making models from human's perspective. We do not know when there will be an error and what causes it in medical images. Medical images reflect on people's health; hence, interpretability is crucial. Now, people often use sensitivity analysis or gradient-based analysis methods for interpretability analysis. There are many attempts to implement interpretability after training such as surrogate models, knowledge distillation, and hidden layer visualization.

RETRACTED

#### 4.3.3. Resolution and Processing of Data Imbalance

Data imbalance often occurs due to inconsistent machine models in medical image segmentation. But in fact, many common imbalance problems can be avoided. Nowadays, the common ways to solve them include expanding the data, using different evaluation indicators, resampling the data set, trying artificial data samples, and using different algorithms. It was suggested in a recent ICML paper that the increased amount of data could increase the error of the training set with a known distribution and destroys the original training set's allocation, thereby improving the classifier's performance. This paper implicitly used mathematical methods to increase the data without changing the size of the data set. However, we believe that destroying the original distribution is beneficial for dealing with imbalances.

#### 4.3.4. A New Exploration of Transformer and Attention Mechanism

This paper introduced attention and transformer methods that afford an innovative combination of these two mechanisms and U-Net. So far, some research has explored the feasibility of using the Transformer structure which only works on the self-attention mechanism as an encoder for medical image segmentation without any pretraining. In the future, more novel models will be proposed to solve different problems in medical segmentation with continuous breakthroughs in attention and transformer methods.

#### 4.3.5. Multimodal Learning and Application

Single-modal representation learning is to express information as numerical vectors that could be processed by the computer or further abstracted into higher-level feature vectors, while multimodal representation learning is to eliminate intermodality by taking advantage of the complementarity between multiple modalities. In medical images, multimodal data with different imaging mechanisms could provide information at multiple levels. Multimodal image segmentation is used to fuse information among different modalities for multimodal fusion and collaborative learning. Research on multimodal learning is becoming more popular in recent years and the application of medical images will grow more sophisticated in the future.

## 5. Discussion and Conclusion

This paper introduces several classic networks with improved U-Net structures to deal with different problems that are encountered in medical image segmentation. We review the paper.

RETRACTED

A summary of the technical context based on the U-Net extended structure introduced above is shown in Figure 7.

This paper summarized U-Net network dimensions, improved structure, and structure parameters, along with kernel size.  Table 2 summarized these aspects.

U- Net could meet the high-precision segmentation of all lesions with its differentiation of organ structures and the diversification of lesion shapes. With the development and improvement of attention mechanism, dense module, transformer module, residual structure, graph cut, and other modules, different modules based on U-Net have been used recently to achieve precise segmentation of different lesions. Based on the various U-Net extended structures, this paper classifies and analyzes several classic medical image segmentation methods based on the U-Net structure.

It is concluded that U-Net-based architecture is indeed quite ground-breaking and valuable in medical image analysis. However, although U-Net-based deep learning has become a dominant method in a variety of complex tasks such as medical image segmentation and classification, it is not all-powerful. It is essential to be familiar with key concepts and advantages of U-Net variants as well as limitations of it, in order to leverage it in radiology research with the goal of improving radiologist performance and, eventually, patient care. Despite the many challenges remaining in deep learning-based image analysis, U-Net is expected to be one of the major paths forward [72–80].

## Figures and Tables

**Figure 1:** Illustration of relative rates of imaging for United States compared with Ontario from year 2000 to year 2016. CT indicates computed tomography; MRI indicates magnetic resonance imaging. All US data are shown as solid curves; Ontario data are shown as dashed curves [1]. (a) All examinations. (b) CT. (c) MRI. (d) Ultrasound.

**Figure 2:** Illustration of U-Net convolution network structure. The left side of the U-shape is the encoding stage, also called contraction path with each layer consisting of two 3 ∗ 3 convolutions with ReLu activation and a 2 ∗ 2 maximum pooling layer. The right side of the U-shape, also called expansion part, consists of the decoding stage and the upsampling process that is realized via 2 ∗ 2 deconvolution to reduce the quantity of input channels by half [2].

**Figure 3:** The U-Net model structure of the proposed AG is added. The input image is gradually filtered and downsampled at each scale in the network's encoding part (for example, H4 = H1/8), indicating the quantity of classes. The gates (AGs) filter the characteristics of propagation by skipping connections. The feature AGs is selected by extracting context information (gating) from a coarser scale [8].

RETRACTED

**Figure 4:** CE-net network structure diagram. (a) The original U-Net encoder block is first supplemented by the ResNet-34 block, shown as (b), to be pretrained by ImageNet. A dense convolution (DAC) block and a RMP block were contained in the bottleneck module. Eventually, the features are withdrawn and gathered in the decoder module. The feature size is enlarged by a decoder block (c), including 1 × 1 convolution and 3 × 3 deconvolution operations, to supplement the original upsampling operation [11].

**Figure 5:** A graphic overview of UNet, UNet++, and UNet 3+. By optimizing jump connections and using full-scale depth monitoring, UNet 3+ integrates multiscale features and produces more precise location perception and segmentation maps with clarified boundaries, regardless of the fewer parameters provided [14, 46].

**Figure 6:** Overview of TransUNet's framework. (a) The transformer layer's structure and (b) the entire TransUNet's structure. After the U-Net encoding stage of the network, a transformer structure composed of 12 layers of transformers is added to process the corresponding processed image sequence. Then the number of channels and dimensions of the picture are unified to the standard by redetermining the size [17].

**Figure 7:** U-Net-based extension structure summary diagram.

**Table 1:** Performance contrast of the networks listed in this article. Different methods use different data sets for evaluation, which makes it hard to compare various approaches horizontally.

U-net type	Medical image data base	Evaluation parameters	Values
U-Net [1]	DRIVE [1]	Accuracy	0.955 ± 0.003 [1]
	Amazon data set	IoU	0.9530 [64]

3D U-Net [29]	Xenopus kidney embryos	IoU	0.732 [29]

Attention U-Net [7]	Gastric cancer [7]	Dice coefficient	0.767 ± 0.132 [7]
	Amazon data set [64]	IoU	0.9581 [64]

CE-Net [10]	DRIVE [10]	Accuracy	0.975 ± 0.003 [10]
	Lung segmentation CT	IoU	0.9495 [65]

U-Net++ [12]	Cell nuclei [12]	Jaccard/IoU	0.9263 [12]
	Lung segmentation CT [65]	IoU	0.9521 [65]

UNET 3+ [13]	ISBI LiTS 2017	Dice coefficient	0.9552

nnU-Net [14]	BRATS challenge	Dice coefficient	0.8987 ± 0.157

U2 Net [15]	Vienna reading [15]	Dice coefficient	0.8943 ± 0.04 [15]
	CVC-ClinicDB	IoU	0.8611 [66]

TransUNet [16]	MICCAI 2015	Dice coefficient	0.7748
	CVC-ClinicDB	IoU	0.89 [66]

**Table 2:** The summary of the changes in network structures and adjusted parameters. The number of parameters for a *K* × *K*(×*K*) size convolution kernel, *C*_*i*_ input channels, and *C*_*o*_ output channels is a *K* × *K*(×*K*) × *C*_*i*_ × *C*_*o*_ and is given below for a few U-Net variants.

Model structure	Dimension	Improved structure	Highlights	#Params	Kernel size
U-Net	2D	Fully connected layer (relative to CNN)	Fully connected layer changed to upsampling layer	30M [67]	3 × 3; 2 × 2; 1 × 1
3D U-Net	3D	Encoder, decoder	2D convolution operation replaced with 3D	19M [68]	1 × 1 × 1; 2 × 2 × 2; 3 × 3 × 3
Attention U-Net	2D	Skip connection	Add the attention module to the skip connection	123M [65]	1 × 1
CE-Net	2D	Bottleneck between encoder and decoder	DAC and RMP structure	110 [65]	3 × 3; 1 × 1
UNET++	2D	Skip connection	Use dense blocks and in-depth supervision	35 [65]	3 × 3; 1 × 1
UNET 3+	2D	Skip connection	Full-scale jump connection and deep supervision	26.97 [69]	3 × 3; 3 × 3 × 3
nnU-Net	2D/3d	Network organization	Multiple ordinary U-Nets form a network pool		4 × 4 × 4
U2-Net	2D	Encoder and decoder	Use RSU as the decoding and encoding unit	176M [70]	3 × 3
Trans-U-Net	2D	Encoder	Add the transformer module after the decoder	2.93M [66, 71]	1 × 1
